The article "Research on Mental Health Education Model of College Students under the Background of Internet" was retracted in 2023. Reasons: signs of a paper mill; suspected computer-generated content; unreliable results or conclusions; concerns about the data.

# Research on Mental Health Education Model of College Students under the Background of Internet

**DOI:** 10.1155/2022/9979891

**Published:** 2022-04-18

**Authors:** Xiaoxin Xia

**Affiliations:** Maanshan Technical College, Maanshan 243000, Anhui Province, China

## Abstract

With the development of information technology, the Internet has been integrated into our life. The psychological education of college students, as the most active group in cyberspace, tends to be diversified, and they will inevitably face various psychological puzzles and conflicts. In order to improve the effectiveness of mental health education in colleges and universities in the network age, colleges and universities use the network platform to build online education mode, which has achieved initial results. This paper analyzes the development status of college students' mental health education in the Internet age, studies its existing problems and challenges, explores its future development trend, expounds the advantages of developing it, and puts forward the main strategies for strengthening it. In order to meet these challenges, college teachers should improve their cognition, constantly explore and develop in practice, actively introduce modern information technology, and give full play to the role of campus culture, so that mental health education can be smoothly carried out in schools.

## 1. Introduction

The construction of a network education platform brings new ideas for college students' mental health education and also makes the traditional education mode face new challenges. The implementation of education reform is also increasing due to the increasing competition faced by college students, college students' learning, and psychological pressure. It is very important to strengthen college students' mental health education, which is of great value to the current social stability, campus stability, and economic development. With regard to mental health, the research report said that college students are facing pressure related to college entrance, and depressive symptoms are one of the most frequently reported mental health problems among this group. At the same time, if students' self-discipline level is not high, the relatively free and independent living space of the university will increase the use of the Internet, which will have a negative impact on physical and mental health. How to carry out effective mental health education for college students in the Internet age is a topic worthy of study. College students' talents have become an important foundation for national development, and the mental health of college students has attracted more and more attention from all walks of life. As a new educational tool, the application of network in mental health education needs the correct guidance of teachers, plays the positive role of network mainstream thought, alleviates the dilemma of current mental health education, and provides theoretical and technical help for the development of college students' positive psychological quality and healthy personality. Many university and college students' mental health education systems in China have made some achievements in education, but the research results of system construction in college students' mental health education are very scarce. The development of Internet technology in the education industry provides a new platform for the development and progress of education and teaching, which especially and fully meets the requirements of college students' mental health education. With the increase of online psychological science resources, it was more convenient and authoritative to use the Internet for psychological education [1]. There are risks of overestimation or underestimation in diagnosing individual's mental health. It is unsure whether the mental health diagnosis system based on DSM is reliable and effective (Davies and Bhugra) [2]. They may be restored to mental health step by step without intervention (Greenspoon and Saklofske, 2001; Keyes, 2007; Suldo and Shaffer, 2008) or obtain mental health by increasing individual's positive forces (Dunn and Dougherty, 2005) [3,4]. At present, most local undergraduate universities in China have adopted various ways to actively educate college students about mental health, such as offering mental health courses, psychological counseling centers, and psychological counseling hotlines. In the configuration of educational facilities and instruments, there are a variety of activity rooms, training rooms, decompression rooms, and psychotherapy and psychological relaxation instruments to relieve the pressure of teachers and students in the whole school and provide material basis for promoting mental health [5]. From a certain point of view, the application of Internet technology in college students' mental health education can lay a solid foundation for the construction of college students' healthy psychology by optimizing the methods and environment of college students' mental health education. However, the mental health education activities carried out by some colleges and universities have not achieved the expected results and failed to give full play to the strategic value of mental health education activities. In this case, it is necessary for educators to conduct a comprehensive and in-depth exploration of the management mode of mental health education for college students.

## 2. Method

### 2.1. Analysis of Internet Technology Forms Commonly Used in Psychological Education

At present, many colleges and universities adopt the “one-stop” mental health education service supermarket [6] when implementing mental health education. As a website, the “one-stop” mental health education service supermarket mainly integrates various disciplines and theories, so that students can use various organs to master psychological knowledge and seek suitable ways to vent and improve their psychological problems through communication with others. Essentially, the “one-stop” website of mental health education service supermarket is the way for students to learn and improve their mental health education knowledge.

Through the analysis of the construction goal, design requirements, and storage network automatic service platform of “one-stop” mental health education service supermarket, the present situation of the model construction of school Internet technology platform is fully grasped, and the matters needing attention in the platform construction are pointed out. The core content of the participatory network mutual assistance platform under the service supermarket is “emphasizing participation.” With the help of the network mutual aid platform, college students can fully communicate with others on this platform and effectively realize mutual assistance [7].

In college students' mental health education, there are many forms of application of Internet technology. Using Internet technology to interact with computer network platforms is a common form [8]. On the auxiliary platform, college students can make friends on the Internet platform through QQ, WeChat, NetEase, and other chat tools, thus greatly reducing their sense of loss and inferiority. During the period of mental health education, college teachers can strengthen the collection of college students' information and establish students' mental health records. On this basis, teachers can conduct comprehensive evaluation and classification according to the psychological characteristics and cognitive status of college students and establish dynamic monitoring systems for different students.

On the basis of fully studying and thinking, perfecting system transformation and theory, this paper discusses the needs of college students' mental health education. When establishing the education system, we should form a multilevel comprehensive education system, actively play the role of grass-roots counselors and student cadres, establish a targeted overall framework of preventive mental health education, and improve the basic goal of university mental health level. The distribution of mental health management in some colleges and universities is shown in Figure 1.

According to the characteristics of students' mental health education framework, we establish a multilevel learning model, such as the full implementation of school-higher education construction. Through expert lectures and personal interviews, students' cognition of family problems and other problems is solved, and then factors that may lead to students' educational crisis are screened out, so as to avoid the impact of social problems on college students' psychology.

In view of the mental health education model of college students, it is necessary to pay full attention to the key issues in students' learning process, so as to establish a comprehensive mental health education and prevention system without missing or concentrating on “points.” Combined with self-help, we establish multilevel crisis intervention model and plan, pay attention to the later work, and minimize the psychological problems caused by the crisis. With the help of pictures, words, music, animation, images, etc., combined with case teaching method, lectures on mental health knowledge, and other professional courses, the knowledge of college students' mental health education books is made into vivid teaching courseware, enriching the forms of mental health education for college students and creating a more relaxed and harmonious learning atmosphere [9].

### 2.2. Application Advantages of Psychological Health Education in Internet Era

At present, in the process of combining network with mental health education, it has the characteristics of times, convenience and transcending time and space. Network mental health education is a new way of social mental health. With the technical support of the Internet, mental health education is characterized by interactivity, diversity, and autonomy.

In the Internet age, information-based psychological education is characterized by fast communication efficiency and high degree of information openness. Establishing psychological intervention education mode on the network platform can expand offline teaching activities and help educators and psychological counselors to change their ideas in time and actively carry out psychological education.  Figure 2 is the flow chart of mental health statistics on the Internet. The network integrates a large number of mental health education resources, expands the information base of mental health knowledge, enriches the knowledge of mental health education, and meets the information needs of students.

The rational introduction of network technology in college students' psychological education can accurately understand the dynamic changes of students' thoughts, grasp the perplexities and problems of students, provide timely guidance and intervention, prevent students from forming psychological problems, and make “student-oriented” thinking become the fundamental principle of psychological intervention. College students' networking and communication can increase the scope of students' communication, break the limitations of traditional communication, make communication more direct and effective, and help college students to establish good psychological quality. For example, at present, the more common services like Post Bar, Weibo, e-mail, etc. enable students to give full play to their thoughts and opinions on the network communication platform, break the limitation of status in traditional communication, make everyone equal in the process of network communication, provide a communication platform for people who are introverted and have insufficient language expression ability in real life, and promote their interpersonal communication. They can also ensure that the society can fully tap the talents of college students, give full play to the true value of college students, and promote social development and progress.

Contemporary college students' psychological problems are increasing day by day, with complex types and distinct characteristics of the times. Communication through the Internet has the function of anonymity, which is economical, convenient, and time-sensitive. This can not only reduce college students' concerns about privacy disclosure, enhance their sense of security, and make them more willing to share their experiences and try to actively contact psychological counselors, but also enable college students to actively contact psychological counseling that suits them according to their own wishes. At the same time, it can also reduce the shyness of college students, make the communication in consultation more possible, and get more information about visitors' self-perception. Adaptability to environmental changes helps students get the methods to maintain mental health and improve their psychological quality, so that students can self-regulate their emotions, face any difficulties alone, and self-regulate and show their perfect self. Huang Hai, Yan Xiaoyong, Yu Li, Yu Zonghuo, etc. pointed out in “college students' attitude towards online psychological counseling and its relationship with personality and network self-efficacy” that college students have a positive attitude towards online counseling. It provides a platform for ideological exchange and interpersonal communication for the majority of students, especially those who are introverted, shy of talking, and weak in social skills [10]. It breaks through the limitations of realistic mental health education.

The network has the advantages of novelty, equality, and strong interaction, which accords with the characteristics of college students' psychological development, and is conducive to stimulating college students' interest and enthusiasm, making them change from “passively accepting knowledge” to “actively participating in” learning, thus enhancing students' learning effect. Analyzing students' information such as browsing online psychological knowledge, watching online psychological videos, conducting online psychological evaluation, and receiving online psychological consultation will help teachers to accurately grasp the psychological trends of college students, educate and guide college students in a timely manner, and intervene and help students with psychological problems. The function of psychological education is to cultivate students' ability to resist pressure. In addition, mental health education can improve students' learning efficiency and teach students more effective learning methods. At the same time, it can cultivate students' innovative thinking and ability to put it into practice, so that students will not be at a loss in the process of interpersonal communication, can communicate with people around them more easily, and can better adapt to the social environment.

### 2.3. Problems in College Students' Mental Health Education

College students have more and more opportunities to access network information. College students who live in the network environment for a long time are easily influenced by bad information. Even if they are found by teachers, it does not matter, which will affect their mental health in the long run. For some introverted and insecure students, they urgently need to find spiritual sustenance through the Internet. However, the temptation and trap on the Internet are everywhere, and students lack enough social experience, so they are easily influenced by the bad information on the Internet, thus endangering their physical and mental health.

Contemporary college students are facing various problems in study, employment, interpersonal relationships, economy, and so on, and their learning competition is becoming increasingly fierce. The emergence of these factors is earlier than now. These factors appeared earlier than now because the environment for college students to grow up has become more complex, the campus environment is no longer the simple model of the past, and changes in social rhythms make schools change rapidly. College students' mental health education still faces multiple dilemmas, including the negative impact of bad information on students, the imperfect construction of online education platforms, and the conflict between personalized education and teaching efficiency. These problems have become the dilemma of college students' growth and development.

There are too many uncertainties in the network. In the Internet age, to carry out network teaching, it is necessary to have multimedia, campus network, and other basic conditions, but many schools have not invested enough in mental health education, and the basic equipment has not been perfect. In college students' mental health education, the application of Internet technology as a new form of education requires teachers to have the good educational professional ability. Only when teachers have sufficient Internet technology teaching ability, can we ensure reasonable and accurate education and teaching for students, improve the teaching quality of college students' mental health education, and improve the adaptability of students' Internet technology teaching.

The most obvious limitation of college students' mental health education is the contradiction between individuality and efficiency. For example, although the general courses and psychological counseling activities of college students' mental health education have a large audience at one time and high overall efficiency, there are inherent limitations in solving individual psychological problems and the quality of individual mental health education. In contrast, the establishment of the psychological counseling room is inefficient and takes a lot of time although it has advantages in solving individual specific problems. Besides, whether it can play its role mainly depends on the initiative of college students.

College students' mental health education platform is not perfect in the following aspects:

University administrators do not pay enough attention to the construction of online education platform. A perfect online teaching platform can provide teachers with a more convenient teaching environment and enable students to acquire mental health knowledge in a relaxed and pleasant environment. However, as a matter of fact, at present, university administrators have not invested funds, manpower, and material resources in the construction of the network platform, nor have they perfected the management system of the network platform; thus, relevant teaching equipment cannot be used by teachers and students.

There is a lack of policy support for the construction of online education platform. At present, some government departments have not issued policies for the construction of online education platform, and local colleges and universities cannot be equipped with better teaching platforms, which causes the mental health education platform for college students to still stay in the past stage.

The evaluation content of online education platform is not perfect. At present, when evaluating the effect of mental health education for students in colleges and universities, we find that most of them use offline questionnaires but seldom use online evaluation. In this case, teachers cannot determine whether college students really understand the teaching content of mental health and how well they have mastered it.

### 2.4. Innovative Ways and Strategies of College Students' Psychological Health Education in the Network Era

According to the characteristics of the times, it is the task of the whole society to find ways to solve the psychological problems of college students. In view of the fact that the psychological problems of college students in the Internet age are mainly manifested in theory and practice, they should be considered when seeking solutions. In the process of breaking through from these two dimensions, the responsibility and mission of mental health educators are particularly arduous. Specifically, this paper mainly discusses the innovation of college students' mental health education from three aspects. In view of this new environment and form, according to the social, economic, and political changes and other factors, combined with the characteristics of college students' own growth, the well-explained theory of mental health education should be reformed to better serve the work of frontline workers and better meet the needs of college students' self-development. Strengthening the theoretical research of mental health education in the network age needs the support of the government.

When conducting mental health education, colleges and universities should combine the educational characteristics of their own schools, clarify their educational goals and tasks, unify the teaching objectives of the whole school, put the interests of students first, and make it clear that the obligations of colleges and universities are not only to impart knowledge to students and manage students, but also to provide daily services for students. We should also use WeChat official account to establish a daily evaluation platform. Students can give feedback to the school if they have any opinions and suggestions on teachers and courses in their daily life, and colleges and universities should do a good job of daily supervision [11] to cultivate students' positive emotions and potential qualities, improve their psychological quality, and promote all-round physical and mental development [12].

In the new media environment, the downloading and browsing of videos are no longer limited to small platforms but can be disseminated and browsed through the Internet. Specifically, teaching resources can be developed through the web, TV dramas, FM, mobile terminals, and other ways. All-media planning is an essential part of film and television teaching. We should actively adapt to the trend of the times, transform teaching methods and educational concepts, and actively meet the opportunities and challenges brought by the Internet. At the same time, colleges and universities should also take advantage of the opportunities brought by the Internet to actively optimize the faculty of colleges and universities, optimize the allocation of educational resources, use big data to practice the concept of personalized education, and do a good job in the investigation of college students' mental health through the information technology platform, so as to prevent the occurrence of college students' mental diseases, scientifically summarize the new features of college mental health education under the background of the Internet, and accurately grasp the rules of college students' mental health education. Therefore, colleges and universities should build teaching mechanisms from a student-centered perspective, always pay attention to students' mental health, do a good job of investigation and guidance, and safeguard students' mental health [13]. Following the principles of people-oriented, individualized, developmental, and holistic mental health education, we will construct a new model of mental health education for college students from the aspects of educational team, teaching resources, educational ideas, network advantages, etc., so as to improve the mental health level of contemporary college students and promote them to become new generations who can shoulder the great cause of national rejuvenation.

Relying on the management and guidance center of mental health education in the school, based on the mental health counseling studio, and focusing on the class mental health education group, we will build a three-level integrated mental health education system for college students, carry out the psychological mutual assistance activities of online psychological counseling, further play the positive role of peer psychological counseling and counseling, and help students get out of their psychological difficulties [14]. With the core of accelerating the integration of information technology and college students' mental health education and teaching, the new ecology of “Internet + education” will be built in an all-round way to realize the informatization of college students' mental health education. According to this principle, this paper constructs a new model of college students' mental health education from three aspects: online evaluation standard, online psychological consultation platform, and online and offline education integration courses. See Figure 3 for details.

## 3. Results

College students are in a critical period of ideological construction. In the face of complex information and external temptation, they are prone to psychological and ideological problems. Colleges and universities should deeply understand the influence of network on students, use the advantages of network education, establish a sound psychological intervention mechanism, help students distinguish multiple pieces of information, and strengthen their network adaptability. At the same time, mental health educators should combine theoretical content, fully integrate network education resources, carry out psychological education activities through multiple channels, and enrich ideological and ideological guidance. Through online and offline cooperation, they should strengthen psychological guidance and correction effect, help students to build positive psychological quality, and promote all-round development, to achieve the fundamental goal of moral education in colleges and universities under the new education environment. This paper analyzes the development status of college students' mental health education in the Internet age, studies its existing problems and challenges, explores its future development trend, expounds the advantages of developing it, and puts forward the main strategies for strengthening it.

## 4. Conclusion and Discussion

Not only is developing mental health education in colleges and universities an arduous and long-term task, but it also faces many challenges. In order to meet these challenges, college teachers should improve their cognition, constantly explore and develop in practice, actively introduce modern information technology, and give full play to the role of campus culture, so that mental health education can be smoothly carried out in schools. We should combine theoretical content, fully integrate network teaching resources, carry out mental education activities through various channels, and innovate teaching modes in the development. The mental health education of college students cannot be separated from teachers' Internet thinking as well. Specific mental health education needs to be piloted and then adjusted according to students' feedback and [15] opinions. The current exploration of mental health education still has great limitations.

## Figures and Tables

**Figure 1:** Mental health management allocation in some colleges and universities.

**Figure 2:** The flow chart of mental health statistics on the Internet.

**Figure 3:** A new mode of mental health education for college students under the background of the Internet.

## Data Availability

The datasets used and/or analyzed during the current study are available from the author on reasonable request.
